# Cuproptosis Combined with lncRNAs Predicts the Prognosis and Immune Microenvironment of Breast Cancer

**DOI:** 10.1155/2022/5422698

**Published:** 2022-09-29

**Authors:** Liangping Zhang, Yujun Zhang, Jianhang Bao, Wenshuo Gao, Dong Wang, Hao Pan

**Affiliations:** ^1^Zhejiang Chinese Medical University, Hangzhou School of Clinical Medicine, Hangzhou, 310000 Zhejiang Province, China; ^2^Department of Orthopaedics, Hangzhou TCM Hospital of Zhejiang Chinese Medical University (Hangzhou Hospital of Traditional Chinese Medicine), Hangzhou, 310000 Zhejiang Province, China

## Abstract

Breast cancer (BC), the most common cancer in women, is caused by the uncontrolled proliferation of mammary epithelial cells under the action of a variety of carcinogenic factors. Cuproptosis-related targets have been found to be closely associated with breast cancer development. TCGA obtained 1226 tumor samples, 1073 clinical data, and 37 lncRNAs during univariate Cox multivariate analysis. We used nonnegative matrix factoring (NMF) agglomeration to spot thirty-three potential molecular subsets with totally different cuproptosis-related lncRNA expression patterns. The least absolute shrinkage and selection operator (LASSO) formula and variable Cox multivariate analysis were not used to construct the best prognostic model. The variations in neoplasm mutation burden and factor gene ontology (GO) and gene set enrichment analysis (GSEA) within the high- and low-risk teams were analyzed, and therefore, the potential mechanism of the development of carcinoma was analyzed. We created a prognostic profile consisting of nineteen cuproptosis-related genes (NFE2L2, LIPT1, LIPT2, DLD, etc.) and their connected targets. The correlation between tumor mutational burden (TMB) and clinical manifestations of tumors demonstrates the importance of high- and low-expression bunch data on the incidence of clinical manifestations of tumors. The area under the curve (AUC) shows moderate prophetic power for copper mortality. GO enrichment analysis showed that immunorelated responses were enriched. Correlation analysis of immune cells showed that pathology could play an important role in the prevalence and prognosis of tumors, and there were variations in immune cells between the probable and low-risk groups. Our study suggests that the prognostic characteristic genes associated with cuproptosis can be used as new biomarkers to predict the prognosis of breast cancer patients. In addition, we found that immunotherapy may play a key role in breast cancer treatment regimens. Levels of immune-associated cells and pathways vary significantly among risk groups of breast cancer patients.

## 1. Introduction

With the improvement in medical treatment, the death rate for breast cancer has dropped dramatically [1, 2]. A range of treatments have been developed to combat the onset and progression of cancer, such as brachytherapy for treating various malignancies [3] and local breast surgery for metastatic breast cancer [4]. RNA therapy for breast cancer plays a significant regulatory role in cell-targeted therapy by increasing or silencing the expression of specific proteins [5] and includes emerging immunotherapy strategies, such as intratumoral therapy and antitumor vaccines [6]. Despite the rapid development of treatments, sometimes, a single treatment fails to achieve the desired effect. Moreover, for triple-negative breast cancer, which is more likely to relapse and metastasize and has a low survival rate, there are a lack of clear targets and limited therapeutic interventions [7]. Therefore, it is particularly important to find more effective therapeutic schemes and regulatory targets for breast cancer. In cancer development and progression, long noncoding RNAs play a crucial role [8]. It has been found that the long noncoding RNA Neat1 promotes growth and metastasis of breast cancer in some studies [9]. In triple-negative breast cancer (TNBC), long noncoding RNAs (lncRNAs) increase invasion, migration, tumor growth, and decrease apoptosis [10]. There has been evidence that abnormally expressed lncRNAs are associated with poor prognoses in TNBC tissues. Due to these specific characteristics, lncRNAs have emerged as novel diagnostic and prognostic biomarkers for TNBC treatment.

We know that the nucleus contains copper and that cancer cells contain higher levels of copper than normal cells, but the mechanisms are poorly studied, and the functional significance of more copper and the underlying mechanisms are still poorly understood [11]. Copper metabolism-related targets have been reported as potential breast cancer therapeutic targets, since they stimulate angiogenesis and metastasis and are essential to cell proliferation and survival [12]. The main method of cuproptosis depends on the buildup of living copper ions. Copper ions directly bind to the lipoacylated elements of the TCA cycle, resulting in the aggregation and disorder of those proteins and blocking the TCA cycle, thus leading to macromolecule cytotoxic stress and death [13, 14]. FDX1 is a key regulator of cuproptosis and an upstream regulator of protein lipoylation [15]. For breast cancer patients, immunotherapy cannot be ignored, and immune checkpoint blockade therapies have been used in a variety of cancers [16, 17]. Metals are known to be important for metabolic activity; however, once excess metals exceed the flexibility of cells to bind inert compounds, they become toxic [18, 19]. Some data mining studies of cancer patients have shown upregulation of the mitochondrial copper-chaperone and cochaperone proteins COX17 and SCO2 [20]. The regulatory mechanism of the copper-related pathway is important for breast cancer development.

In this study, we hope to find a completely unique lncRNA feature that can accurately predict the prognosis of tumor patients, and at the same time, we will analyze the possible role of cuproptosis-related lncRNA as a tumor therapeutic target to find a key signaling pathway for the treatment of breast cancer.

## 2. Materials and Methods

### 2.1. Collection and Grouping of Breast Cancer Data

The RNA-sequencing and clinical data of The Cancer Genome Atlas (TCGA) BRCA dataset were downloaded from TCGA (https://tcga-data.nci.nih.gov/tcga/). The cohort consisted of 1098 carcinoma patients with relevant organic phenomenon profiles and clinical characteristics, and 25 patients were then excluded because of incomplete transcriptomic and clinical information. The remaining data with complete follow-up information (*n* = 1073) was included in our dataset for more analysis.

### 2.2. Analysis of High and Low lncRNA Expression Groups

First, we distinguished lncRNAs from total RNA. Through correlation analysis, we obtained cuproptosis-related lncRNAs, and univariate Cox regression analysis was applied to obtain lncRNA-related prognoses. Moreover, the downloaded carcinoma samples were divided into 2 groups in a step with the expression level of lncRNAs through nonnegative matrix factorization (NMF) clustering, namely, the lncRNA high-expression cluster and the lncRNA low-expression cluster. Heat maps of the high expression cluster and therefore the low expression cluster were used to analyze the correlation of clinical manifestations of the samples. Then, the ESTIMATE algorithm and CIBERSORT were applied to analyze the differences in the immune microenvironment (stromal score, immune score, ESTIMATE score, and tumor purity) and immune cell infiltration between group 1 and group 2.

### 2.3. Construction of the Model and the Nomogram

The least absolute shrinkage and selection operator (LASSO) and multivariate Cox regression analyses are used in this analysis; we obtained a prognostic model based on 16 lncRNAs. At the same time, heat maps were drawn to show the expression in 1073 patients. Furthermore, to predict the prognosis more efficiently, a nomogram was used. Before the nomogram, we ran univariate Cox regression and multivariate Cox regression analysis to determine which clinical characteristics could be used as an influential factor.

### 2.4. Tumor Mutation Analysis

In the model, patient groups with high-expression breast cancer and those with low-expression breast cancer showed a difference. The gene mutation burden of groups with high expression was calculated. Mutation counts were clearly observed in both the high-expression and low-expression groups, and the relationship between mutations and risk was investigated.

### 2.5. Functional Enrichment Analysis

Using differentially expressed genes (DEGs) of the different levels of risk groups, we ran gene ontology (GO) to identify potential pathways. GO analysis showed significant enrichment of immune-related molecules. They included body substance immune reactions, modulating cell surface receptor signal pathway substances, and receptor-mediated signal pathway immune reactions.

### 2.6. Immune Cell Infiltration and Immune Function Analysis

Based on the GO results, we explored more immune-related studies. CIBERSORT was used to calculate the abundance of immune cells, and a single-sample gene set enrichment analysis (ssGSEA) was used to compare immune function between different levels of risk individuals. A gene set enrichment analysis (GSEA) was performed to analyze the differences in pathways between the two groups.

### 2.7. Statistical Analyses

R (version 4.2.0 https://cran.r-project.org/bin/windows/base/) and Perl (version 5.30.0.1; https://www.perl.org/get.html) programming languages were used to extract and process clinical information and RNA sequences. The cutoff value for differentially expressed FRGs was set at ∣log_2_fold change | >0.5, and a false discovery rate (FDR) < 0.05 was used. The *t* test and chi-square test were used to calculate whether the results were significantly different.

## 3. Results and Discussion

### 3.1. Nonnegative Matrix Factorization (NMF) Clustering

It can be seen from the figure that there were differences between high-expression clusters and low-expression clusters (Figures 1(a) and 1(b)). High lncRNA expression clusters showed significant differences in ESTIMATE score, immune score, stromal score, and tumor purity atmospheres. The ESTIMATE score of high-expression cluster patients was significantly higher than one of low expression cluster patients (Figure 1(c)), and the immune score of high-expression cluster patients was significantly higher than one of low-expression cluster patients (Figure 1(d)). The stromal score of the patients with high expression was significantly higher than that of the patients with low expression (Figure 1(e)), and tumor purity was significantly lower in patients with high expression than in patients with low expression (Figure 1(f)). We compared the high expression and low expression of lncRNA, indicating important variations in tumor-infiltrating immune cells between the risk cluster and the low-risk cluster. Comparing the two groups shows that there is a difference in the proportion of infiltrating immune cells (Figure 1(g)). There were differences in immune cell content and the microenvironment between patients with high lncRNA expression and patients with low-risk lncRNAs, so there was a high correlation between immune cells (Figure 1(h)).

### 3.2. Analysis of High- and Low-Expression lncRNA Immune Cells

To check the variations in infiltrating immune cells between the risky and low-risk teams, a box diagram was made. The proportion of resting memory CD4 T-cells, naive B-cells, and resting mast cells in the risky cluster was considerably higher than that in the low-risk cluster. The proportion of T helper cells in the risk cluster was higher than that in the low-risk cluster (Figure 2).

### 3.3. Cuproptosis Genes Associated with Breast Cancer Have Significant Prognostic Value

Thirty-seven related lncRNAs were used as the prediction model (Figure 3(a)). A correlation heat map was used to show the DEG correlations associated with cuproptosis. (Figure 3(b)). LASSO multivariate analysis was used to validate the model (Figure 3(c)). Risk scores in different levels of risk clusters were distinguished by heat maps (Figure 3(d)). Univariate results showed that the model scores were different except for gender, and multivariate results showed that the model scores and age regional units were different in high-risk and low-risk groups (Figures 3(e) and 3(f)).

### 3.4. Construction and Evaluation of the Gene Prognosis Model in TCGA

Similarly, it is possible to predict patient survival based on the risk score (Figure 4(a)), and the area under the curve (AUC) confirmed that the identified prognostic characteristics predicted BRCA survival (AUC = 0.766, 0.808, and 0.745; 1 year, 2 years, and 3 years (Figure 4(b)), while other scoring methods had a higher concordance index (Figure 4(c)). By building a prognostic model, patients can be scored according to their age, gender, clinical stage of tumor, and other conditions, and the 1-3 year survival rate of patients can be predicted (Figure 4(d)).

### 3.5. Clinical Manifestations of the Low-Risk and High-Risk Groups

The prognostic model was used to further study patients according to tumor stage, age, sex, and so on as the classification. Differences in tumor stages and ages were observed between the high- and low-expression groups. The high-risk patient survival rate and survival rate were significantly lower than those of the low-risk patients (Figure 5).

### 3.6. Different Stemness Statuses in the Low-Risk and High-Risk Groups

PCA was used to analyze the BCSC-associated lncRNA risk model, a comparison of 19 cuproptosis-related coding genes and genome-wide expression profiles between different risk individuals (Figures 6(a) and 6(b)). In the risk model, there were different distribution directions between the different risk groups (Figures 6(c) and 6(d)), indicating that the risk model can divide breast cancer patients into two parts, and the situation of different levels of risk patients is different. Based on the survival rate and progression-free survival rate, with further functional annotation, the risk model of related genes in the breast cancer group and the survival rate of differentially expressed genes between different levels of risk patients showed differences in the survival rate of different levels of risk patients during the dry correlation process. The survival rate of the high-risk group was relatively low, and the survival rate of the high-risk group was relatively low (Figure 6(e)). Prognostic values of risk models associated with lncRNAs in TCGA cohort were evaluated. The Kaplan-Meier survival analysis was performed for different levels of risk patients based on the risk model and median risk score. Based on the risk score, breast cancer patients were divided into different risk levels, and the median risk score was determined. Kaplan-Meier survival analysis showed a lower overall survival in high-risk patients than in low-risk patients (Figure 6(f)). In an attempt to explain the relationship between risk scores and survival of breast cancer patients, risk curves and scatter plots were used. Risk scores are correlated with mortality rates (Figures 6(g) and 6(h)).

### 3.7. Independent Validation of Mutations

In the two groups of patients with a genetic mutation burden calculation, it was clearly observed that in patients with breast cancer, significantly higher mutation counts and high mutation rates were observed in the high-expression and low-expression groups. In the high-risk group of patients with low risk and with high and low mutation samples, the mutation of counting was visible, with PI3CA, TP53, and TTN genes being prone to light mutations, such as Frame_Shift_Del and Missense_Mutation (Figures 7(a) and 7(b)). In the risk models, there were differences in tumor mutation burden (Figure 7(c)), and patients in the low-risk group had a significantly lower survival rate than those in the high-risk group (Figure 7(d)). The survival rates of the high mutation group of patients and the high-risk group of patients were lower than those of the low mutation group and the low-risk group of patients (Figure 7(e)); thus, the prediction model in the high-risk groups for breast cancer survival prediction was statistically significant.

### 3.8. Immune-Related Functions and Pathways Are Enriched in GO

GO analysis showed significant enrichment of several immune-related molecules. These included the humoral immune response, regulation of cell surface antigens of receptor signaling pathways, receptor-mediated immune response signal channels, activation of the signal transduction of the immune response, activation of cell surface receptor signaling pathways of circulating immune globulin mediating the humoral immune response, activation of the B-cell activation of complement activation of the immune response, B-cell receptor signaling pathways, and other related immune pathways (Figures 8(a) and 8(b)).

### 3.9. The Immune Cell Infiltration Landscape in Breast Cancer

In further exploration of the relationship between ferroptosis and breast cancer-related lncRNAs and antitumor immunity, tumor-infiltrating immune cells were found to be significant in both groups. The correlation matrix of the proportion of all tumor-infiltrating immune cells is shown in Figure 9(a). The differences in different immune cells, such as timer, CIBERSORT, CIBERSORT−ABS, and QUANTISEQ, can be seen in the heat map of immune cells (Figure 9(b)). B-cells, CD8+ T-cells, and DC scores in the low-risk group were significantly lower than those in the high-risk group (Figure 9(c)). Comparison of immune function showed that the scores of cytolytic activity, HLA, and inflammatory function in the low-risk group were significantly lower than those in the high-risk group (Figure 9(d)). A low-risk group had lower levels of PDHA1, DLD, NLRP3, and other immune checkpoint molecules than a high-risk group (Figure 9(e)).

### 3.10. Correlations Were Identified by Gene Set Enrichment Analysis (GSEA)

Biological functions and signal transduction pathways of lncRNAs related to cuproptosis and differentially expressed cistrons in bad and low-risk teams were used for gene set enrichment analysis (GSEA). The results showed that in bad carcinoma patients, the expression of cell cycle, complement and natural action cascade, cytokines, and protein receptor interactions was upregulated. The expression of the JAK STAT signaling pathway was significantly downregulated (Figure 10).

### 3.11. Discussion

In recent years, the incidence of breast cancer has been increasing [21], and people are also looking for more effective diagnosis and treatment plans. With an increasing number of treatment plans for breast cancer, we know that many lncRNAs play a critical role in the development of cancer [22]. For example, lncRNAs can inhibit the progression of colorectal cancer by activating YAP [23]. lncRNAs promote liver cancer tumor growth by regulating mir-154/PCNA/HBV cccDNA signal transduction and HBV replication [24]. lncRNAs can regulate metabolism in cancer [25, 26]. lncRNAs regulate intracellular and extracellular-derived metabolism, thereby influencing the behavior of cancer cells and regulating the tumor microenvironment [27, 28]. Long noncoding RNA (lncRNA) also shows its regulatory role in cancer drug resistance [29]. In the past decade, RNA-based therapeutics have gained considerable clinical attention, mainly through the use of antisense oligonucleotides and small interfering RNAs [30]. Unfortunately, so far, no clinical trials have been conducted with lncRNA therapeutics. The role of long noncoding RNAs as biomarkers is actively being explored, confirming their prevalence as disease markers.

There is growing evidence that copper metabolism is a key factor in promoting breast cancer [31, 32]. The immune system is closely related to copper metabolism. In cancer cells, copper supplements enhance the expression of pD-L1 at both mRNA and protein levels. Copper modulates key signaling pathways that control PD-L1-induced cancer immune escape and promote mediated degradation of PD-L1. Interestingly, copper chelating agents increased tumor-infiltrating CD8 T-cells and natural killer cells and slowed tumor growth [33]. It may therefore be possible to change copper metabolism and improve immune function by regulating copper metabolism-related lncRNAs. Meanwhile, improving copper metabolism may be an effective strategy for breast cancer treatment. In our study, we identified 37 copper metabolism-related lncRNAs associated with breast cancer prognosis. The proportion of resting CD4 T-cells, naive B-cells, and resting mast cells was inhibited in the high-risk group. In our study, consensus clustering of 37 prognostic lncRNAs showed that the two clusters were higher in the group with high expression of the ESTIMATE score, immune score, and stromal score lncRNA and lower in the group with high expression of neoplasm lncRNA. We know that the immune score is a biomarker for estimating overall breast cancer survival that is associated with important immunophenotypic factors and that patients with high immune scores exhibit therapeutic benefits from chemotherapy and immunotherapy [34]. Univariate Cox regression and LASSO Cox regression analyses were used to construct a copper metabolism-related lncRNA profile, including 19 copper metabolism-related lncRNAs. In our study, this feature was shown to be a good predictor of overall survival, mutation burden, immune-related function, and immunotherapy response in different levels of risk breast cancer groups. A rosette was constructed to analyze the likely 1-, 3- and 5-year overall survival rates of patients with breast cancer [35]. It can be seen from our study that the area under curve and AUC confirmed the prognostic characteristics and predicted the survival of BRCA. The consistency index of other scoring methods was higher. Differences in tumor stage and age were significant between the different levels of risk groups, and risk scores could be used as predictors.

Immunity is essential to the treatment of tumors. In the established clinical prediction model for carcinoma, the GO enrichment analysis of differential genes within the high- and low-risk teams showed that the biological processes were concentrated in immune response−activated cell surface receptor signaling pathway, circulating immunoglobulin mediated by humoral immune response, B-cell complement-activated immune response activation, and B-cell receptor signaling pathway. The cell components were enriched in immunoglobulin complex, immunoglobulin complex, and the immunoglobulin complex pathway by molecular enrichment. It is known that the immune pathway is widely activated. In our study, patients at low risk of breast cancer had a higher tumor mutation burden, and it is known that a high tumor mutation burden (TMB) can benefit immunotherapy across multiple tumor types [36]. The study found that the tumor mutation burden and specific immune cells were associated with the response, and B-cell T follicular-assisted cell activation promoted the antitumor response [37]. In our study, the T-cell CD4 memory resting group, the B-cell naive group, and the mast cell resting group were significantly lower than the low-risk group. Certain immune cells are more active in a low-risk mutation burden. Consistent with the established model, lncRNAs associated with ferroptosis play a vital role in immune regulation. In our study, GSEA was enriched in the cell cycle pathway. We know from the diagram that the cell cycle pathway is upregulated in the high-risk group. Immunity is closely related to the cell cycle [38], which has extensive immunomodulatory effects mediated by CDK4/CDK6 inhibitors in the different levels of risk groups [39]. We know that autophagy directly eliminates microbes inside cells [40]. In addition, the relationship between neutrophils and circulating tumor cells regulates cell cycle progression in the blood and increases the metastatic potential of circulating tumor cells [41, 42]. The expression of the high-risk JAK STAT signaling pathway was significantly downregulated. JAK_STAT was enriched in the different levels of risk groups. The JAK/STAT signaling is a common intracellular signaling pathway that regulates cell apoptosis and the immune system [43]. In tumorigenesis, maintenance, and metastasis, JAK/STAT signaling plays an important role [44, 45]. Further experiments are needed to validate the pathway analysis between the different levels of risk groups.

Our study has some limitations. First, our study relies on TCGA public information, and this cuproptosis-related lncRNA prognostic model needs further validation using prospective, multicenter, real-world data. Second, our study preliminarily discovered the connection between cuproptosis-related lncRNAs and antitumor immunity. The underlying mechanism must be further explored through additional experiments.

## 4. Conclusion

In conclusion, we found cuproptosis-related gene that may accurately predict the prognosis of carcinoma patients. The current study observed that it could be used to classify patients with BRCA according to their respective clinical and molecular features. The novel prognostic model could independently predict the risk associated with the survival of patients with BRCA in the derivation and validation cohorts, which indicated a strong predictive value. Patients with high risk scores may experience an adverse immune environment and have poor clinical outcomes. lncRNAs related to cuproptosis could play a possible role in growth immunity and become therapeutic targets for carcinoma. Through our studies, we found that the JAK_STAT signaling pathway may be an important pathway involved in immune regulation. The potential mechanisms and their biological functions in BRCA and cuproptosis -related genes remain unclear and warrant further research.

## Figures and Tables

**Figure 1:** (a) The samples were divided into 2 groups in keeping with the high and low expression of lncRNA. (b) The clinical connectedness of heat map and lncRNA expression between the 2 groups. (c) ESTIMATE score. (d) Immune score. (e) Stromal score. (f) Neoplasm purity. (g) Percentage of infiltrating immune cells. (h) Immunocell correlation diagram in cluster.

**Figure 2:** Analysis of immune-related differences between the two groups. (a) T-cell regulatory (Treg) comparison between the two subgroups. (b) T-cell comparison between the two subgroups. (c) T-cell CD4 memory resting between the two subgroups. (d) T-cell CD8 between the two subgroups. (e) T-cell CD4 memory activated between the two subgroups. (f) TNK-cell activated comparison between the two subgroups. (g) Mast cell resting comparison between the two subgroups. (h) Macrophage M0 comparison between the two subgroups. (i) B-cell naive comparison between the two subgroups.

**Figure 3:** (a) Forest map of 37 CuPro-related lncRNAs. (b) Heat map of the correlation between lncRNA and cuproptosis-related targets. (c) A prognostic risk prediction model was constructed. (d) lncRNA heat map of the different levels of risk groups. (e–f) Seven clinically relevant forest maps were analyzed by univariate Cox regression.

**Figure 4:** (a) Clinically relevant ROC curve of the model. (b) 1-3 year ROC curve of the model. (c) *C*-index curve of 7 clinical factories. (d) Nomogram score and clinical characteristics.

**Figure 5:** Survival risk scoring model. (a, b) Survival rate of patients in the medium-high risk group with different tumor stages. (c) Survival rate of women in the medium-high risk group. (d, e) Survival rate of patients in different age groups with high and low risk. (f, g) Survival rate of patients in the low-medium risk groups with different T stages of tumor tissue. (h, i) Survival rate of patients in the medium-high risk groups with different N stages of tumor tissue.

**Figure 6:** (a) PCA of all genes. (b) Different risks of cuproptosis-related genes. (c) Different risks of cuproptosis-related lncRNAs. (d) Different risks of lncRNA expression PCA. (e) The model predicted survival in different risks. (f) The model predicted progression-free survival in different risks. (g, h) Risk score distribution and survival status of breast cancer patients in different risks.

**Figure 7:** Analysis of mutation burden in breast cancer samples. (a, b) Waterfall diagram of gene mutations in samples from the groups of different risks. (c) Relationship between tumor mutation burden in samples from the groups of high-low risk. (d) Relationship between survival rate in the high-low mutation burden group. (e) Relationship between survival rate in the high-low mutation burden group and the high-high risk group.

**Figure 8:** An analysis of gene ontology (GO) visualizing biological processes, molecular functions, and cellular components enriched by DEGs (a, b).

**Figure 9:** Analysis of immune-related functional differences based on GO analysis results. (a) Immune cell map of the sample. (b) Immune-related heat map. (c) Map of immune cells in the groups of different risks. (d) Map of immune function in the groups of different risks. (e) Map of immune checkpoints.

**Figure 10:** GSEA pathway was different between the high- and low-expression groups. (a) Cell cycle. (b) Chemokine signaling pathway. (c) JAK_STAT signaling pathway. (d) Complement and coagulation cascades. (e) Basal transcription factors. (f) Cell adhesion molecules.

## Data Availability

All raw data of the expression level and clinical information of patient samples are downloaded from TCGA database (https://portal.gdc.cancer.gov/), which is a publicly available database.

## Supplementary Materials

Supplementary Materials 137 differentially expressed genes.

## References

[1] Wojtyla C., Bertuccio P., Wojtyla A., La Vecchia C. (2021). European trends in breast cancer mortality, 1980-2017 and predictions to 2025. *European Journal of Cancer*.

[2] DeSantis C. E., Ma J., Goding Sauer A., Newman L. A., Jemal A. (2017). Breast cancer statistics, 2017, racial disparity in mortality by state. *CA: a Cancer Journal for Clinicians*.

[3] Deng X., Wu H., Gao F. (2017). Brachytherapy in the treatment of breast cancer. *International Journal of Clinical Oncology*.

[4] Tosello G., Torloni M. R., Mota B. S., Neeman T., Riera R., Cochrane Breast Cancer Group (2018). Breast surgery for metastatic breast cancer. *Cochrane Database of Systematic Reviews*.

[5] Song Y., Ke X., Chen L. (2021). The potential use of RNA-based therapeutics for breast cancer treatment. *Current Medicinal Chemistry*.

[6] Huppert L. A., Mariotti V., Chien A. J., Soliman H. H. (2022). Emerging immunotherapeutic strategies for the treatment of breast cancer. *Breast Cancer Research and Treatment*.

[7] Zhu Y., Zhu X., Tang C., Guan X., Zhang W. (2021). Progress and challenges of immunotherapy in triple-negative breast cancer. *Biochimica Et Biophysica Acta. Reviews on Cancer*.

[8] Liu S., Sun Y., Hou Y. (2021). A novel lncRNA ROPM-mediated lipid metabolism governs breast cancer stem cell properties. *Journal of Hematology & Oncology*.

[9] Park M. K., Zhang L., Min K. W. (2021). _NEAT1_ is essential for metabolic changes that promote breast cancer growth and metastasis. *Cell Metabolism*.

[10] Thakur K. K., Kumar A., Banik K. (2021). Long noncoding RNAs in triple-negative breast cancer: a new frontier in the regulation of tumorigenesis. *Journal of Cellular Physiology*.

[11] Chen L., Li N., Zhang M. (2021). APEX2-based proximity labeling of Atox1 identifies CRIP2 as a nuclear copper- binding protein that regulates autophagy activation. *Angewandte Chemie (International Ed. in English)*.

[12] Karginova O., Weekley C. M., Raoul A. (2019). Inhibition of copper transport induces apoptosis in triple-negative breast cancer cells and suppresses tumor angiogenesis. *Molecular Cancer Therapeutics*.

[13] Tsvetkov P., Coy S., Petrova B. (2022). Copper induces cell death by targeting lipoylated TCA cycle proteins. *Science*.

[14] Cobine P. A., Brady D. C. (2022). Cuproptosis: cellular and molecular mechanisms underlying copper-induced cell death. *Molecular Cell*.

[15] Tsvetkov P., Detappe A., Cai K. (2019). Mitochondrial metabolism promotes adaptation to proteotoxic stress. *Nature Chemical Biology*.

[16] Blockhuys S., Celauro E., Hildesjo C. (2017). Defining the human copper proteome and analysis of its expression variation in cancers. *Metallomics*.

[17] Masoumi E., Tahaghoghi-Hajghorbani S., Jafarzadeh L., Sanaei M. J., Pourbagheri-Sigaroodi A., Bashash D. (2021). The application of immune checkpoint blockade in breast cancer and the emerging role of nanoparticle. *Journal of Controlled Release*.

[18] Cobine P. A., Moore S. A., Leary S. C. (2021). Getting out what you put in: copper in mitochondria and its impacts on human disease. *Biochimica Et Biophysica Acta (BBA)-Molecular Cell Research*.

[19] Tang D., Chen X., Kroemer G. (2022). Cuproptosis: a copper-triggered modality of mitochondrial cell death. *Cell Research*.

[20] Chen J., Jiang Y., Shi H., Peng Y., Fan X., Li C. (2020). The molecular mechanisms of copper metabolism and its roles in human diseases. *Pflügers Archiv*.

[21] Ahmad A. (2019). Breast cancer statistics: recent trends. *Advances in Experimental Medicine and Biology*.

[22] Peng W. X., Koirala P., Mo Y. Y. (2017). LncRNA-mediated regulation of cell signaling in cancer. *Oncogene*.

[23] Ni W., Yao S., Zhou Y. (2019). Long noncoding RNA GAS5 inhibits progression of colorectal cancer by interacting with and triggering YAP phosphorylation and degradation and is negatively regulated by the m^6^A reader YTHDF3. *Molecular Cancer*.

[24] Feng J., Yang G., Liu Y. (2019). LncRNA PCNAP1 modulates hepatitis B virus replication and enhances tumor growth of liver cancer. *Theranostics*.

[25] Tan Y. T., Lin J. F., Li T., Li J. J., Xu R. H., Ju H. Q. (2021). LncRNA-mediated posttranslational modifications and reprogramming of energy metabolism in cancer. *Cancer Communications*.

[26] Chi Y., Wang D., Wang J., Yu W., Yang J. (2019). Long non-coding RNA in the pathogenesis of cancers. *Cells*.

[27] Lin W., Zhou Q., Wang C. Q. (2020). LncRNAs regulate metabolism in cancer. *International Journal of Biological Sciences*.

[28] Sun Z., Yang S., Zhou Q. (2018). Emerging role of exosome-derived long non-coding RNAs in tumor microenvironment. *Molecular Cancer*.

[29] Luo Y., Zheng S., Wu Q. (2021). Long noncoding RNA (lncRNA)EIF3J-DTinduces chemoresistance of gastric cancer via autophagy activation. *Autophagy*.

[30] Winkle M., El-Daly S. M., Fabbri M., Calin G. A. (2021). Noncoding RNA therapeutics -- challenges and potential solutions. *Nature Reviews. Drug Discovery*.

[31] Ramchandani D., Berisa M., Tavarez D. A. (2021). Copper depletion modulates mitochondrial oxidative phosphorylation to impair triple negative breast cancer metastasis. *Nature Communications*.

[32] Laws K., Bineva-Todd G., Eskandari A., Lu C., O'Reilly N., Suntharalingam K. (2018). A copper(II) phenanthroline metallopeptide that targets and disrupts mitochondrial function in breast cancer stem cells. *Angewandte Chemie (International Ed. in English)*.

[33] Voli F., Valli E., Lerra L. (2020). Intratumoral copper modulates PD-L1 expression and influences tumor immune evasion. *Cancer Research*.

[34] Wang S., Zhang Q., Yu C., Cao Y., Zuo Y., Yang L. (2021). Immune cell infiltration-based signature for prognosis and immunogenomic analysis in breast cancer. *Briefings in Bioinformatics*.

[35] Bandos A. I., Rockette H. E., Song T., Gur D. (2009). Area under the free-response ROC curve (FROC) and a related summary index. *Biometrics*.

[36] Barroso-Sousa R., Jain E., Cohen O. (2020). Prevalence and mutational determinants of high tumor mutation burden in breast cancer. *Annals of Oncology*.

[37] Hollern D. P., Xu N., Thennavan A. (2019). B cells and T follicular helper cells mediate response to checkpoint inhibitors in high mutation burden mouse models of breast cancer. *Cell*.

[38] Goel S., DeCristo M. J., Watt A. C. (2017). CDK4/6 inhibition triggers anti-tumour immunity. *Nature*.

[39] Petroni G., Formenti S. C., Chen-Kiang S., Galluzzi L. (2020). Immunomodulation by anticancer cell cycle inhibitors. *Nature Reviews. Immunology*.

[40] Kuo C. J., Hansen M., Troemel E. (2018). Autophagy and innate immunity: insights from invertebrate model organisms. *Autophagy*.

[41] Szczerba B. M., Castro-Giner F., Vetter M. (2019). Neutrophils escort circulating tumour cells to enable cell cycle progression. *Nature*.

[42] Hidalgo A., Chilvers E. R., Summers C., Koenderman L. (2019). The neutrophil life cycle. *Trends in Immunology*.

[43] Xin P., Xu X., Deng C. (2020). The role of JAK/STAT signaling pathway and its inhibitors in diseases. *International Immunopharmacology*.

[44] Shao F., Pang X., Baeg G. H. (2021). Targeting the JAK/STAT signaling pathway for breast cancer. *Current Medicinal Chemistry*.

[45] Tabassum S., Abbasi R., Ahmad N., Farooqi A. A. (2019). Targeting of JAK-STAT signaling in breast cancer: therapeutic strategies to overcome drug resistance. *Advances in Experimental Medicine and Biology*.

